The article "To Explore the Haemostatic Effect of Compression Haemostasis Using an Ultrasonic Probe under the Guidance of Ultrasound after Radial Artery Puncture" was retracted in 2023. Reasons: signs of a paper mill; suspected computer-generated content; unreliable results or conclusions; lack of ethics approval or compliance.

# To Explore the Haemostatic Effect of Compression Haemostasis Using an Ultrasonic Probe under the Guidance of Ultrasound after Radial Artery Puncture

**DOI:** 10.1155/2021/7423101

**Published:** 2021-12-01

**Authors:** Xianwei Jin, Qiaoling Weng, Jia Min

**Affiliations:** ^1^Department of Anesthesiology, The First Affiliated Hospital of Nanchang University, 17 Yong Wai Zheng Street, Nanchang, Jiangxi 330006, China; ^2^Department of Anesthesiology, The Second Affiliated Hospital of Nanchang University, Nanchang University, No. 1, Minde Road, Nanchang City Jiangxi 330008, China

## Abstract

**Objective:**

To evaluate a new haemostasis method using an ultrasound probe to compress the radial artery and haemostasis under direct vision to replace traditional manual compression of the radial artery.

**Methods:**

According to a random number table, 240 patients with gastrointestinal tumours who had undergone arterial puncture were divided into Group A (120 cases) and Group B (120 cases). In Group A, patients were under the guidance of ultrasound to confirm the vascular port, determine the compression position of the ultrasound probe, observe the degree of vascular deformation, and press the radial artery puncture port with pressure to stop bleeding under direct vision. In Group B, traditional manual compression was used. All patients received 5 min of compression for haemostasis, and haemostasis conditions were recorded after compression and 24 hours postoperatively.

**Results:**

The incidence of bleeding, haematoma, and skin ecchymosis at the puncture site after 5 minutes of compression in Group A was lower than that in Group B (*P* < 0.05). No significant difference was found between the two groups at 24 hours after the operation (*P* > 0.05).

**Conclusion:**

The method using an ultrasound probe to guide radial artery compression to haemostasis is better than traditional manual compression when applied for compression haemostasis after removing the radial artery catheter.

## 1. Introduction

With advances in medicine, an increasing number of complex patients and surgical methods appear in the clinic. Among these methods, arterial puncture has become particularly important. Radial artery catheterization is generally used for haemodynamic monitoring and internal environment analysis [1, 2] and is the most common choice for arterial catheter placement. The complications of radial artery puncture has always been an unavoidable problem and can be divided into puncture-staged complications [3–6] and catheterization removal-staged complications [7, 8]. Presently, studies on reducing the complications of arterial puncture domestically and abroad have primarily focused on interventional surgery [9–12]. Few studies have investigated routine arterial puncture used to monitor vital signs. Compared with the interventional surgery, the daily puncture volume is large, and the removal of the arterial puncture catheter is the final process of the entire radial artery puncture process. Determining the severity of complications after arterial puncture is also crucial. Clinically, no unified guidance exists regarding how to better stop bleeding after removing radial artery puncture catheters. Although the incidence of corresponding complications is not high, because of the large number of punctures, its absolute number is not small, and the potential adverse impacts on the postoperative rehabilitation of patients should be considered.

With the advances in ultrasound technology for arterial puncture, complications in the arterial puncture stage are reduced [13, 14]. However, the application of ultrasonic probes in radial artery puncture mostly occurs in the puncture stage [15–17]. Few studies have investigated the extraction stage of radial artery catheters. The application of compression haemostasis using an ultrasonic probe has been used in the previous nonsurgical treatment of iatrogenic femoral artery pseudoaneurysms [18–20]. Capewell et al. studied the haemostatic effect of manual compression of the radial artery using different operators as early as the 1990s [21]. It is obvious that ultrasound has not been fully recognized for its value in this process. During ultrasound-guided arterial puncture, the angle between the puncture needle and the skin and the variation degree of the artery itself cause that the puncture point where the needle tip enters the blood and the puncture point displayed on the skin may not be on the vertical line perpendicular to the pressing direction of the arm [22]. In a study of 505 patients, Valsecchi et al. found that 22.8% of patients exhibited anatomical variation of the upper limb artery, and the tortuosity of the radial artery reached 3.8% [23]. The benefit of ultrasonic probes for compression haemostasis after extubation of the radial artery is predictable. Therefore, the present study investigated the use of an ultrasonic probe to guide postoperative radial artery catheterization removal and explore the value of this technology in compression haemostasis after removing radial artery puncture.

## 2. Data and Methods

### 2.1. Clinical Data

From June 2021 to August 2021, 240 patients aged 17-82 years had undergone radial artery catheterization and postanesthesia care unit (PACU) resuscitation and extubation at the First Affiliated Operating Room of Nanchang University. The inclusion criteria were as follows: patients with 20G arterial catheterization for invasive arterial pressure monitoring; a negative Allen test—the same puncture site was punctured only once [24]; and no bleeding, haematoma, or ecchymosis on the skin at the puncture site. The exclusion criteria were as follows: bleeding and haematoma during puncture catheterization; a history of subcutaneous puncture bleeding or peripheral vascular diseases before this puncture; an abnormal platelet count; and abnormal coagulation function. Regarding exclusion and shedding, cases that did not meet the inclusion criteria or did not stop bleeding according to the predetermined scheme after inclusion as required were excluded. During implementation, a case in which the patient did not cooperate or withdraw personally was regarded as shedding. Using the random number table method, 240 patients who had met the inclusion criteria were randomly divided into 120 cases in the experimental group (Group A) and 120 cases in the control group (Group B). In Group A, a high-frequency linear array probe, was used to stop bleeding. The specific operation method was to first use the long axis of the high-frequency linear array probe parallel to the arterial direction to identify the arterial puncture point instead of the skin puncture point, turn on the colour blood flow function on ultrasound, and apply appropriate pressure directly above the arterial puncture point using the short axis of the high-frequency linear array probe perpendicular to the arterial direction. During the removal of the arterial puncture catheter and subsequent compression process, the ultrasound should not show overflow of the arterial blood colour blood flow.

### 2.2. Instrument Preparation

Ultrasound was performed using the Navis Compass ultrasound system (China Shenzhen Huasheng Medical Technology Ltd.) and the following additional materials: a 20 G artery puncture needle, a sterile hole towel, a soft tape, sterile gloves, a sterile gauze, a transparent applicator, a disposable aseptic ultrasonic probe protective sleeve, and a medical ultrasonic probe disinfectant gel.

### 2.3. Methods

#### 2.3.1. Radial Artery Catheterization

The Allen test was performed in both groups before the operation, and radial artery catheterization was performed after general anaesthesia. The patients were placed in the supine position, straightening the arm, keeping the palm upwards or relaxing the hand naturally, padding the wrist high, keeping the wrist joint in the hyperextension state, and disinfecting with iodophor. A region with a range of more than 10 cm, whose central point was the position where the radial artery pulsation was strongest at 1 cm from the proximal styloid process of radius, was punctured by the same experienced anaesthesiologist. An anaesthesiologist was required to wear gloves, spread the aseptic hole towel, smear the gel on the high-frequency linear array ultrasonic probe, and cover the aseptic protective sleeve. The frequency range of the ultrasonic probe was maintained at 5~13 MHz, and arterial puncture was performed at an angle of 30~45° between the needle trunk and skin. After connecting the sensor, the puncture needle catheter was fixed with a transparent dressing, and the invasive arterial pressure was monitored after calibration.

#### 2.3.2. Catheter Removal

The catheter was removed under direct vision by ultrasound in the experimental group and according to the traditional method in the control group. Pressurization was performed for 5 min after pulling out the needle [21, 25] by two trained anaesthesia nurses chosen randomly. The control group was treated with traditional manual compression haemostasis: the fixed applicator was removed and disinfected with iodophor cotton swab, centred on the puncture point, with a range larger than 10 cm. The puncture point was covered with twice-folded sterile gauze, the radial artery catheter was removed out, and the skin puncture point was pressed with the finger pulp (Figure 1). For the experimental group, the fixed applicator was removed and the same disinfection method was performed. The colour blood flow function on the ultrasound was turned on, the high-frequency linear array probe was selected, the long axis was made parallel to the direction of the artery, and the artery puncture point was located for the artery puncture needle (Figures 2 and 3). Next, an ultrasonic probe coated with a gel and a sterile protective sleeve were used to locate the puncture needle vascular port. Once the puncture entrance is located, the high-frequency linear array probe was rotated to the short axis perpendicular to the arterial direction. The radial artery catheter was removed and pressed directly above the vessel puncture needle wound under the direct field of vision of the ultrasonic probe (Figures 4–6). After pressing for 5 min, the gauze and ultrasonic probe were removed from the two groups, and the haemostatic effect of pressing was observed. If bleeding continued, the operator would pressurize for another 5 min. Additionally, the compression times were recorded until haemostasis was successful.

### 2.4. Observed Indicators

The observed indicators were as follows: bleeding— bleeding at the skin puncture point visible to the naked eye; subcutaneous haemorrhage; clinical manifestations—ecchymosis (diameter < 2 mm), purpura (diameter: 3~5 mm), ecchymosis (diameter > 5 mm), and subcutaneous haematoma (diameter usually > 10 mm, deep haemorrhage with or without skin uplift) [26, 27]; average perfusion index (Pi) value and its change rate within 10 s before and after compression haemostasis; visual analogue score (VAS) of pain during compression; and times of compression haemostasis. The evaluators were anaesthesiologists who had received unified training. When assessing the results, the conditions of haemostasis in different groups were determined by observation and measurement of skin changes at the puncture point of the radial artery. The measurements were performed in strict accordance with standard operation.

### 2.5. Sample Capacity and Statistical Analysis

According to our preliminary studies, the expected incidence of bleeding in Group A was 5%, while that in Group B was 17.5%. Assuming that the type I error is 0.05 and the efficacy is 0.80, the calculated sample capacity of the study is at least 194 individuals. Considering that some patients may be eliminated because of changes in clinical conditions, 240 patients were initially recruited for the study. Categorical data were expressed as numbers or percentages, and quantitative data showing a normal distribution were expressed as means and standard deviation. Chi-squared test and Fisher probabilities were used to analyse categorical data. *P* < 0.05 was considered the statistically significant critical point. All the data were analysed by SPSS.

## 3. Results

### 3.1. Comparison of the General Conditions of the Two Patient Groups

No significant difference was found between the groups in age, sex, height, weight, platelet value, mean arterial pressure, heart rate, oxygen saturation decrease value, arterial condition, or other general conditions (*P* > 0.05) (Table 1).

### 3.2. Comparison of Changes in Vital Signs during Compression between the Patient Groups

The average change rates of Pi values during compression haemostasis in Group A and Group B were 5.725% and 33.225%, respectively (*P* < 0.05). The average pressing times of Group A and Group B were 1.058 and 1.291, respectively (*P* < 0.05). The average compression pain VAS scores of Group A and Group B were 1.291 and 2.033, respectively (*P* < 0.05). All data were statistically significant (Table 2).

### 3.3. Effects of Compression Haemostasis on the Two Patient Groups

The incidence rates of bleeding in Group A and Group B were 5.83% and 19.16%, respectively (*P* < 0.05), the incidence rates of haematoma in the two groups were 4.16% and 17.5%, respectively (*P* < 0.05), and the incidence rates of ecchymosis in the two groups were 5% and 14.16%, respectively (*P* < 0.05). All data were statistically significant (Table 3).

## 4. Discussion

Compared with the traditional manual compression group, the incidence of bleeding or subcutaneous hematoma was lower in the ultrasonic probe compression group after radial artery extubation. The success rate of compression haemostasis was higher, revealing that this ultrasound-guided method was effective. The times of compression haemostasis, change rate of Pi and pain severity, which are related, decreased significantly. These secondary results also reflect the reliability of ultrasonic probes for radial artery compression haemostasis.

During compression haemostasis, the pain VAS of the ultrasonic probe pressing group was significantly lower than that of the control group (*P* < 0.05). Good experience brings patient cooperation, which is more conducive to haemostasis. Additionally, the decrease in PI [28, 29] related to peripheral blood perfusion during compression was significantly lower than that in the control group (*P* < 0.05), further indicating that the ultrasonic probe under direct vision can be used to compress the radial artery without affecting the blood supply of the hand. During the compression process of the traditional manual pressing group, the Pi value fluctuates greatly, and the stability is worse than that of the ultrasonic probe pressing group, which may be caused by the uneven force of the operator or sliding on the pressing point. Without visual reference indices, surgery can only be performed based on experience, possibly leading to an unstable haemostasis process and prolonged haemostasis time. At the same time, the times of compression haemostasis in the ultrasonic probe pressing group were also significantly lower than those in the control group (*P* < 0.05). The success rate of ultrasonic probe compression was higher. Most patients can stop bleeding at one time by ultrasonic probe compression. Although the success rate of the traditional manual compression group is not low, as long as the first haemostasis is unsuccessful, more failures will follow. The operator generally suspects that the power of compression is insufficient, thus increasing the compression strength, which increases the difficulty of operation and decreases the degree of Pi. This time-consuming and laborious pressing method, which is difficult for both operators and patients, may affect the formation of platelet haemostatic suppository and blood coagulation and eventually lead to the extension of haemostatic time.

Scientifically solving the postoperative complications of removing radial artery intubation is an urgent problem. Improper operation may cause many complications. Excessive local pressure and a prolonged operation time can cause distal limb ischaemia and even necrosis. However, excessively loose compression can cause bleeding, haematoma formation, pseudoaneurysm, and infection based on haematoma formation [30, 31]. The ultrasonic probe used in this study can easily solve these problems. It has been widely used in nonsurgical compression treatment of iatrogenic pseudoaneurysms because of its cost-effectiveness and reliable haemostatic effect without influencing the blood supply of the hands [32–34]. Similarly, compared with many imprecise and expensive compression haemostasis equipment, the compression haemostasis process can be performed using ultrasound equipment commonly used in the clinic. It is comfortable, portable, low cost, visible, and controllable in the whole process, and the effect is accurate. Therefore, it can be widely used in postoperative radial artery hemostasis.

However, this study has some limitations. First, we selected patients with normal coagulation function and excluded patients with abnormal coagulation function. Thus, the reference value for patients with abnormal coagulation function was missing, warranting further studies in patients with abnormal coagulation function. Second, the analysis of the Pi value only compared the change rate of each patient before and after compression. Many factors can influence the Pi value. The study only assessed the change trend of finger blood perfusion ability without strictly analysing the Pi value before and after compression in Group A and Group B. Finally, differences were found in the evaluation of the patients' pain VAS scores. Trauma operations and the pain threshold of patients are inconsistent, likely affecting the pain score. Additionally, the degree of postoperative wakefulness of patients may affect the accuracy of the pain VAS score.

## 5. Conclusion

Ultrasonic probe-guided radial artery compression haemostasis is better than the traditional manual compression method after removing radial artery catheterization.

## Figures and Tables

**Figure 1:** In the traditional manual pressing haemostasis group, the operator takes the bleeding point of the skin as the pressing point and use his fingers to press haemostasis in the whole process.

**Figure 2:** The long axis of the ultrasonic probe is parallel to the artery.

**Figure 3:** The vascular inlet of the arterial catheter is located when the long axis of the ultrasonic probe is parallel to the artery.

**Figure 4:** The short axis of the ultrasonic probe is perpendicular to the artery.

**Figure 5:** Before pressing haemostasis, the short axis of the ultrasonic probe is perpendicular to the entrance of the arterial puncture needle, and the ultrasonic image is formed at the moment of removing the catheter.

**Figure 6:** Before pressing haemostasis, the short axis of the ultrasonic probe is perpendicular to the arterial puncture needle into the vascular port. After pulling out the catheter, use the ultrasonic probe to press haemostasis with the force that does not show arterial blood flow overflow on the ultrasonic display screen.

**Table 1:** Comparison of the general conditions of the two patient groups.

Group	Experience group (*n* = 120)	Control group (*n* = 120)	*χ* ^2^/*t*	*p*
Age	59.40 ± 12.31	62.09 ± 10.96	-1.788	0.075
Height (cm)	162.59 ± 7.38	163.29 ± 6.41	-0.784	0.434
Weight (kg)	59.28 ± 11.14	60.15 ± 10.54	-0.622	0.535
Platelet value	222.07 ± 49.27	227.67 ± 54.02	-0.839	0.402
Mean arterial pressure	92.14 ± 10.38	91.75 ± 10.07	0.290	0.772
Heart rate	71.28 ± 6.03	70.57 ± 5.97	0.914	0.362
Oxygen saturation (%)	96.85 ± 1.64	96.68 ± 1.81	0.745	0.457
Gender				
Male	78	74	0.287	0.592
Female	42	46		

**Table 2:** Comparison of related indexes during compression haemostasis between the two groups.

Group	Experience group (*n* = 120)	Control group (*n* = 120)	*t*	*p*
Change rate of pi	5.72 ± 2.06	33.22 ± 19.36	-15.465	1.661 × 10^−30^
Times of compress	1.05 ± 0.23	1.29 ± 0.59	-3.968	1.110 × 10^−4^
VAS	1.29 ± 0.45	2.03 ± 1.20	-6.288	3.232 × 10^−9^

**Table 3:** Comparison of hemostatic effect between two groups after compression haemostasis.

Group	Experience group (*n* = 120)	Control group (*n* = 120)	*χ* ^2^	*p*
Bleeding	7/120 (5.83%)	23/120 (19.16%)	9.752	0.002
Haematoma	5/120 (4.16%)	21/120 (17.5%)	11.042	0.001
Ecchymosis	6/120 (5%)	17/120 (14.16%)	5.818	0.016

## Data Availability

All data generated or analysed during this study are included in this published article.
